The article "MiR-140 targets RAP2A to enable the proliferation of insulin-treated ovarian granulosa cells" was retracted in 2023. Reasons: duplicated images; signs of a paper mill; unreliable results or conclusions.

# MiR-140 targets RAP2A to enable the proliferation of insulin-treated ovarian granulosa cells

**DOI:** 10.1186/s13048-020-0611-4

**Published:** 2020-02-05

**Authors:** Zhengfang Xiong, Bing Li, Wenjuan Wang, Xianghui Zeng, Binye Li, Shengyan Jian, Liyun Wang

**Affiliations:** 1 Reproductive Medical Center, Qinghai Provincial People’s Hospital, No. 2, Gonghe Road, Xining, 810007 Qinghai China; 2 Department of General Surgery, Qinghai Provincial People’s Hospital, Xining, 810007 Qinghai China

**Keywords:** Polycystic ovarian syndrome, Ovarian granulosa cells, miR-140, RAP2A, AKT

## Abstract

**Background:**

We elucidated the role of specific MicroRNAs (miRNAs) in the development of polycystic ovary syndrome (PCOS) and explained the changes in the proliferation of granulosa cells. Excised ovarian cortex specimens were collected for miRNA profiling analysis (*n* = 20 PCOS females and 5 non-PCOS females). Insulin-treated ovarian granulosa cells isolated from mice were used for mechanical studies.

**Results:**

High miR-140 expression was observed in PCOS samples and insulin-treated granulosa cells compared to that in non-PCOS and unstimulated cells, respectively. However, the Ras-related protein Rap-2a precursor (RAP2A) was downregulated in in PCOS. MTT assay and EdU staining showed that an miR-140 inhibitor attenuated viability in insulin-treated granulosa cells; cell viability increased with miR-140 overexpression. Reduced expression of miR-140 and the expression of the miR-140 mimic resulted in marked cell apoptosis, as evidenced by the results of PI flow cytometry and Annexin V-FITC; miR-140 overexpression results in downregulated RAP2A expression, and the miR-140 mimic directly bound to the RAP2A 3′-UTR, causing increase in RAP2A levels in insulin-treated granulosa cells; RNA-mediated silencing of RAP2A in insulin-treated granulosa cells restored cell proliferation and apoptosis to normal levels. Phosphorylated AKT was found to be negatively regulated through cross-talk between miR-140 and RAP2A.

**Conclusions:**

In conclusion, PCOS ovarian cortex specimens and insulin-treated granulosa cells showed elevated expression of miR-140, which could lead to increased proliferation and reduced apoptosis of cells by targeting RAP2A. This study may pave the way for future research on the properties of granulosa cells in PCOS.

## Background

At present, nearly 5–10% of all women of childbearing age have been diagnosed with polycystic ovary syndrome (PCOS) [1]. Ultrasound scan results reveal that this disorder is characterized by chronic anovulation, polycystic ovaries, and hyperandrogenemia [2]. PCOS has been regarded as a chief cause of anovulation-induced infertility. Several genetic factors have been reported to explain its etiology; however, no clear conclusions have been reached [3].

The article "MiR-140 targets RAP2A to enable the proliferation of insulin-treated ovarian granulosa cells" was retracted in 2023. Reasons: duplicated images; signs of a paper mill; unreliable results or conclusions.

MicroRNAs (miRNAs) are small (~ 22–25 nucleotide long), non-coding RNAs that regulate the expression of target mRNA transcripts (post-transcriptional gene silencing) [4]. Many studies have highlighted the critical influence of miRNAs on multiple biological processes, such as cell proliferation and the metastasis of malignant tumors. Besides malignancies, numerous processes involved in PCOS pathogenesis (proliferation, differentiation, etc.) also show varied expression of specific miRNAs. Hossain et al. found a positive correlation between the pathogenesis of PCOS and the expression profile of miRNAs in rat ovaries [5]. They used dihydrotestosterone (DHT) to induce PCOS in a rat model; significant differential expression of 25 miRNAs was found between the ovaries of normal and PCOS rats. In DHT-treated ovaries, most of the miRNAs that promoted cyst formation were found to be expressed in the follicular theca cells. It was also found in the PCOS ovaries that miRNA alterations were associated with the dysregulation of molecular pathways. Hyperinsulinemia is one of the most common features of PCOS, therefore, previous studies utilized insulin treatment to recapitulate PCOS in cell models [6–9]. Jiang et al. showed that there is increased expression of miR-93 in PCOS granulosa cells, in which both cell cycle progression and proliferation were promoted by targeting CDKN1A. The expression of miR-93 was upregulated, and cell proliferation was promoted in the insulin-stimulated KGN granulosa cells [10]. In recent years, miR-140 has been reported to exhibit significant regulatory effects with respect to cell proliferation, differentiation, migration, and invasion [11–13]. Scalici et al. showed that the expression of miR-140 in the follicular fluid was different between PCOS and normal ovarian reserves, with a specificity of 83.8% and a sensitivity of 70% [14]. However, the expression profile of miR-140—along with its underlying mechanism during ovarian dysfunction—is still poorly reported. Therefore, more studies are needed to examine the mechanism underlying miR-140-mediated modulation of PCOS.

This study evaluated the effect of miR-140 in the context of PCOS development. The expression of miR-140 in the ovaried of PCOS patient as well as in insulin-stimulated cell lines was evaluated. Moreover, our research also attempted to reveal the effect of miR-140 on cell death in insulin-treated mouse granulosa cells via the RAP2A/AKT axis.

## Results

### miR-140 is upregulated in the ovaries of PCOS patients

The miRNA microarray analysis revealed significant upregulation of miR-140 in PCOS samples (*n* = 6) compared to that in healthy control samples (*n* = 6) (Fig. 1a). To confirm this finding, a qPCR analysis was performed in PCOS specimens and non-PCOS specimens. As opposed to the healthy controls (*n* = 5), PCOS ovaries showed miR-140 upregulation (*n* = 20) (Fig. 1b). We also isolated GCs from 8 PCOS patients and 8 non-PCOS patients to validate the expression of miR-140. The data showed that miR-140 expression was upregulated in the GCs from PCOS patients relative to that in the non-PCOS controls (Fig. 1c). It was presumed that the differences in the expression of miR-140 in our study might be caused by high insulin concentrations, considering the fact that one of the prominent characteristics of PCOS is hyperinsulinemia, and previous studies have utilized insulin treatment to recapitulate PCOS in cell-based models [6–9]. The relationship between insulin stimulation and miR-140 expression was studied in granulosa cells using qPCR. It was found that miR-140 expression increased upon insulin stimulation (Fig. 1d). Thus, miR-140 expression is upregulated in PCOS ovaries.

The article "MiR-140 targets RAP2A to enable the proliferation of insulin-treated ovarian granulosa cells" was retracted in 2023. Reasons: duplicated images; signs of a paper mill; unreliable results or conclusions.

**Fig. 1:** miR-140 expression in ovarian specimens of PCOS subjects and insulin-treated granulosa cells. **a** miRNA microarray showing deregulated miRNAs in ovarian specimens of 6 PCOS patients (PCOS group) and 6 non-PCOS patients (normal group). **b** qPCR analysis confirmed miR-140 expression in the PCOS specimens (*n* = 20) and normal group (*n* = 5). **c** qPCR analysis validated miR-140 expression in human granulosa cells (GC) from PCOS patients (*n* = 8) and non-PCOS patients (*n* = 8). **d** qPCR revealed the miR-140 expression in insulin-treated and untreated GCs. Data represents mean ± SD values from three independent experiments. *P < 0.05 vs. indicated group

### Effect of miR-140 on proliferation and apoptosis of insulin-treated granulosa cells

We measured the expression of miR-140 in insulin-treated granulosa cells to study its role in insulin-treated granulosa cell proliferation (Fig. 2a). An EdU assay was used to explore the role of the varied expression of miR-140 in the cell proliferation of insulin-stimulated granulosa cells. Cell proliferation was greatly reduced after treatment with the miR-140 inhibitor as compared to that in the Normal, Insulin, and NC groups; however, the miR-140 mimic increased cell proliferation (Fig. 2b). Further, the viability of insulin-treated granulosa cells was measured by MTT assay. The miR-140 inhibitor reduced the viability of the granulosa cells while the miR-140 mimic promoted the viability (Fig. 2c, d).

**Fig. 2:** Mediation effect of miR-140 on the viability and apoptosis of insulin-treated granulosa cells. After transfection with miR-140 inhibitor/mimic or NC-inhibitor/mimic, the cells were further treated with a high concentration of insulin (100 ng/ml). **a** qPCR analysis was carried out to detect the miR-140 level in granulosa cells that underwent different treatments. **b** The EdU assay showed miR-140 inhibitor or mimic affected the viability of insulin-treated granulosa cells. **c**, **d** MTT staining was used to determine the proliferation of the insulin-treated granulosa cell proliferation transfected with the miR-140 inhibitor, mimic or their controls. *N* = 3. *P < 0.05, **P < 0.01, ***P < 0.001 vs. indicated group

Afterwards Annexin V-FITC and PI flow cytometry was conducted to investigate the apoptotic level in insulin-treated granulosa cells with varied miR-140 expression. In contrast with the NC and Insulin groups, depletion of miR-140 increased apoptosis while the miR-140 mimic decreased apoptosis in granulosa cells (Fig. 3a, b). Therefore, it can be concluded that miR-140 may protect the insulin-stimulated granulosa cells from apoptosis.

The article "MiR-140 targets RAP2A to enable the proliferation of insulin-treated ovarian granulosa cells" was retracted in 2023. Reasons: duplicated images; signs of a paper mill; unreliable results or conclusions.

**Fig. 3:** Effect of miR-140 on apoptosis of insulin-treated granulosa cells. **a** FC revealed the extent of apoptosis in the differently treated granulosa cells. **b** The histogram shows the level of apoptosis in granulosa cells in response to different treatments. *N* = 3. *P < 0.05 vs. Insulin group

### miR-140 directly targets RAP2A

There is increasing evidence that miR-140 can regulate target genes [15–17]. Bioinformatic analyses have shown that miR-140 may target the 3′-UTR of RAP2A (Fig. 4a). The direct relationship between miR-140 and RAP2A was investigated using DLRA (Fig. 4b). The results showed 80% inhibition of luciferase activity in cells transfected with the WT RAP2A-fixed miR-140 mimic compared to that in control group cells. We also examined RAP2A expression in isolated human GCs. The results showed that RAP2A mRNA expression was reduced in human GCs from PCOS patients (Fig. 4c). Furthermore, for the insulin-stimulated granulosa cells transfected with different products, we also carried out WB and qPCR assays to study the RAP2A expression at the transcriptional and translational levels. We found that the miR-140 inhibitor significantly increased the expression of RAP2A, whereas miR-140 decreased its expression (Fig. 4d, e).

**Fig. 4:** miR-140 targeting of the 3′-UTR of RAP2A. **a** Bioinformatic analysis revealed a miR-140 binding site in the RAP2A gene. **b** DLRA was performed following co-transfection of a luciferase reporter containing either WT (wild-type) or MU (mutant) RAP2A and a miR-140 mimic into HEK293T cells. Data were analyzed with ANOVA with Tukey post-hoc test. *N* = 3. *P < 0.05, **P < 0.01 vs. control group. **c** qPCR analysis validated RAP2A expression in human GC from PCOS patient (*n* = 3) and non-PCOS patients (*n* = 3). **d** qPCR and **e** WB revealed that the RAP2A levels in insulin-treated granulosa cells transfected with miR-140 inhibitor, mimic or their controls. *N* = 3. *P < 0.05, **P < 0.01 vs. indicated group

Further experiments were conducted in the normal group and PCOS group to evaluate miR-140 expression. PCOS specimens showed decreased RAP2A expression compared to that in the controls (Fig. 5a). The RAP2A level in insulin-treated granulosa cells was reduced compared to that in non-treated cells, as evidenced by both WB and qPCR (Fig. 5b, c). Meanwhile, we also found that p-AKT levels showed a reverse trend with respect to RAP2A expression. These data suggest that miR-140 targets the 3′-UTR of RAP2A, while PCOS and insulin treatment of granulosa cells cause a significant reduction in RAP2A.

The article "MiR-140 targets RAP2A to enable the proliferation of insulin-treated ovarian granulosa cells" was retracted in 2023. Reasons: duplicated images; signs of a paper mill; unreliable results or conclusions.

**Fig. 5:** RAP2A expression in PCOS samples and in insulin-treated granulosa cells. **a** qPCR analysis showed decreased RAP2A expression in the ovaries from PCOS patients. **b** The qPCR and **c** WB assays were used to study RAP2A expression in insulin-treated and non-treated granulosa cells at translational and transcriptional levels. *N* = 3. *P < 0.05, **P < 0.01 vs. the indicated group

### RAP2A silencing reversed the effect of miR-140 in insulin-treated granulosa cells

We explored whether RAP2A knockdown could abolish the effects of miR-140 inhibition on insulin-treated granulosa cells. To this end, cells were co-transfected with shRNA-RAP2A/NC and the miR-140 inhibitor. Both qPCR and WB demonstrated that as compared to the RAP2A levels in the Insulin and NC groups, insulin+miR-140 inhibitor+shRAP2A group showed significant downregulation of RAP2A (Fig. 6a). WB also demonstrated that RAP2A inhibition negatively regulated AKT phosphorylation (Fig. 6b, c).

**Fig. 6:** The effect of miR-140 on insulin-treated granulosa cells reversed by the RAP2A inhibitor. Insulin-treated granulosa cells were co-transfected with shRNA-RAP2A/NC and miR-140. **a** qPCR and **b** WB analyses were carried out to evaluate the RAP2A, AKT, and phosphorylated AKT levels in each group. **c** Quantification of phosphorylated AKT. **d** MTT staining was used for determining the proliferation of insulin-treated granulosa cells with different transfections. **e** Flow cytometric analysis showing the extent of apoptosis in the differently treated chondrocytes. **f** Histogram shows the apoptosis level in granulosa cells with different treatments. *N* = 3. *P < 0.05, **P < 0.01, ***P < 0.001 vs. indicated group

The role of RAP2A in the proliferation and apoptosis of cells was also investigated. MTT assay—which was performed in insulin-treated cells co-transfected with shRNA-RAP2A/NC and the miR-140 inhibitor—showed that RAP2A silencing significantly restored the inhibition of cell growth that had been induced by the miR-140 inhibitor (Fig. 6d). Moreover, flow cytometry showed that RAP2A silencing decreased the stimulatory effects of miR-140 inhibition on cellular apoptosis (Fig. 6e, f). Thus, these data suggest that miR-140 could influence the properties of insulin-treated granulosa cells by targeting RAP2A.

The article "MiR-140 targets RAP2A to enable the proliferation of insulin-treated ovarian granulosa cells" was retracted in 2023. Reasons: duplicated images; signs of a paper mill; unreliable results or conclusions.

## Discussion

PCOS is characterized by hyperandrogenism, polycystic ovaries, chronic anovulation, and insulin resistance (IR) [18]. The involvement of miRNAs in the metabolic and biological processes associated with PCOS has been previously reported. In PCOS patients, obesity and the concentration of circulating androgens can influence the expression of miRNA-155, miRNA-103, miRNA-27b, and miRNA-21, and can have a critical impact on metabolic processes [19]. Hossain et al., showed that the theca cells of PCOS subjects showed expression of miR-222 via localization in situ; however, androgens could target P27/kip1 to regulate the proliferation of theca cells, leading to miR-222 repression. Additionally, ERα protein was decreased when the miR-222 was overexpressed, and ERα target gene expression and signaling were also reduced [5]. These results might pave the way for studies on the pathogenesis of PCOS. As evidenced by miRNA expression profiling, Sang et al. reported the crucial effects of a large number of miRNAs on steroidogenesis in the human follicular fluid of PCOS patients. Follicular fluid specimens of patients with PCOS showed significantly decreased miR-320 and miR-132 expression compared to that observed in the control group [20]. Even though miRNA had been indicated to be the key regulator of PCOS [21], there has been an incomplete characterization of miRNA functions in ovarian granulosa cells. Previous studies have demonstrated that miR-140 is a tumor mediator. Song et al. has reported that expression of miR-140 was associated with chemosensitivity in osteosarcoma tumor xenografts. Tumor cells ectopically transfected with miR-140 were more resistant to methotrexate and 5-fluorouracil (5-FU). Overexpression of miR-140 inhibited cell proliferation in osteosarcoma as well as colon cancer cell lines. Histone deacetylase 4 (HDAC4) was confirmed to be one of the important targets of miR-140 [22]. Li et al. found that miR-140 plays a critical role in regulating stem cell signaling in normal breast epithelium and in ductal carcinoma. Moreover, SOX9 and ALDH1—the most significantly activated stem-cell factors in DCIS stem-like cells—are direct targets of miR-140 [16]. Yuan et al. showed that miR-140 is significantly downregulated in human non-small cell lung cancer (NSCLC) tissues and cell lines. Both gain-of-function and loss-of-function studies demonstrated that miR-140 suppresses NSCLC cell proliferation, migration, and invasion in vitro via targeting IGF1R [13]. In colorectal cancer (CRC), miR-140 directly targets Smad2 and overexpression of miR-140 in CRC cell lines results in decrease of Smad2 expression, leading to decreased cell invasion and proliferation, and increased cell cycle arrest [23]. As we mentioned above, miR-140 could regulate multiple genes in different cell lines, in this study, downregulation of RAP2A almost reversed the effect of miR-140 on cell proliferation and apoptosis in insulin-stimulated GCs, suggesting that RAP2A is the dominant target of miR-140 effect in the insulin-treated GCs. In this study, miR-140 was found to be significantly upregulated in the ovaries of PCOS patient and insulin-treated granulosa cells indicating its potential role in PCOS progression. Further study showed that miR-140 depletion caused a noticeable reduction in granulosa cell proliferation. In contrast, the effects were reversed with the transfection of the cells with the miR-140 mimic. Flow cytometry results showed that cellular apoptosis was negatively regulated by miR-140.

The article "MiR-140 targets RAP2A to enable the proliferation of insulin-treated ovarian granulosa cells" was retracted in 2023. Reasons: duplicated images; signs of a paper mill; unreliable results or conclusions.

In the present study, insulin was used to treat GCs in order to establish a PCOS cell model, as one of the most distinct features of PCOS pathogenesis is the insulin-resistance. For this reason, the use of insulin-sensitizers, such as inositol isoforms, gained increasing attention due to their safety profile and effectiveness [24]. Recent data suggests that reduction of insulin levels using diazoxide or insulin sensitizer drugs such as metformin, thiazolidinediones (PPAR-γ agonist), or inositols reduces hyperandrogenism in PCOS [25–27]. Two inositol stereoisomers, myo-inositol (MI) and D-chiro-inositol have been proven to be effective in PCOS treatment. The co-administration of MI and D-chiro-inositol, in the physiological plasma ratio ensures better clinical results, such as the reduction of insulin resistance, androgens’ blood levels, cardiovascular risk, and regularization of menstrual cycle with spontaneous ovulation [28]. Several signal transduction pathways are reported to be involved in insulin resistance, such as peroxisome proliferator-activated receptors (PPARs) [29–31], PI3K, PKC [32], NFκB, and Ras/mitogen-activated protein kinase (MAPK) [33]. Meanwhile, PCOS might be regulated through genetic alterations that activate several signaling pathways, such as the MAPK, PI3K, AKT, ERK1/2, and RAS pathways [29–31, 34–36]. RAP2A belongs to the Ras superfamily, and RAP2A with constitutive activity has been shown to inhibit AKT phosphorylation in B cell lines by binding to PI3K [37]. However, no clear results have been obtained for its function in PCOS. This study showed that the downregulation of RAP2A in insulin-treated granulosa cells increased AKT signaling but had no effect on miR-140 expression (data not shown). The p-AKT level showed a reverse trend with RAP2A expression, which was also reported by Wang et al. [38]. Furthermore, miR-140-induced inhibition of RAP2A contributed to an increase in pAKT, and pAKT expression was significantly restored by RAP2A knockdown. These findings indicate that RAP2A inhibits proliferation and induces apoptosis of insulin-stimulated granulosa cells via downregulation of AKT phosphorylation. Unbalanced proliferation and apoptosis of GCs may lead to abnormal folliculogenesis [39, 40]. Bax is a pro-apoptotic protein, and a recent study has also reported that levels of Bax are significantly upregulated in patients with PCOS when compared with that in healthy controls, indicating that GCs in PCOS patients exhibited a higher incidence of apoptosis than that in healthy controls [41]. A previous study has demonstrated that the transcription factor, p53 is a critical regulator of the cell cycle, DNA repair, and apoptosis, and thet RAP2A is a novel target of p53 and is induced upon DNA damage in a p53-dependent manner [42]. The mouse GC has been widely used to investigate cell growth and apoptosis of human GCs [43]. In this study, miR-140 inhibition significantly promoted apoptosis and inhibited proliferation of GCs, while its overexpression downregulated apoptotic level, thus indicating that miR-140-RAP2A may participate in the pathogenesis of PCOS by inhibiting apoptosis and promoting proliferation of GCs.

The article "MiR-140 targets RAP2A to enable the proliferation of insulin-treated ovarian granulosa cells" was retracted in 2023. Reasons: duplicated images; signs of a paper mill; unreliable results or conclusions.

## Conclusions

In the present study, bioinformatic analysis predicted a presumptive complementary zone of miR-140-RAP2A, which was confirmed by DLRA. The upregulation of miR-140 expression, was found to be negatively correlated with RAP2A expression in insulin-treated granulosa cells. In addition, miR-140 silencing significantly increased RAP2A expression and decreased AKT phosphorylation, and subsequently impacted cell proliferation, while RAP2A silencing restored cell viability in insulin-stimulated granulosa cells. However, the present study utilized a cell-based model to study the mechanism of miR-140 action in the context of PCOS, an animal experimental model should be used in future studies to further confirm the findings of this study. To conclude, our data suggest that in PCOS, miR-140 protects insulin-stimulated granulosa cells from apoptosis by acting as an interceptor of the RAP2A/AKT cross-talk.

## Methods

### Clinical samples

This study was approved by the local research ethics committee of Qinghai Provincial People’s Hospital (Qinghai, China) from where the patients were also recruited. Prior to the experiments, written informed consents were obtained from the subjects. Twenty women with PCOS were undergoing the laparoscopic investigation for infertility. The revised Rotterdam European Society of Human Reproduction for Reproductive Medicine criteria (2003) was used for diagnosing PCOS [44]. Simultaneously, 5 women with normal menstruation and pelvic pain-induced diagnostic laparoscopy, benign condition-induced hysterectomy, and laparoscopic sterilization, were selected as the normal control group. For diagnostic laparoscopy in infertility, biopsy of healthy tissues or lesion tissue was performed. Subsequently, the modified Ferriman-Gallwey score (mFG), hip circumference, waist circumference, weight, height, and other factors were measured. The BMI value was obtained by dividing the body weight in kilograms using height (kg/m^2^). A mechanical, 6-MHz probe-equipped, Toshiba Sonolayer SSA-220A (Toshiba, Tokyo, Japan) was used to conduct the transvaginal ultrasonography for investigating the ovaries. A chemiluminescence immunometric assay, using a commercial kit, was performed to detect the fasting insulin level, and a glucose oxidase assay (Tosoh Corp., Tosoh, Japan) was used for measuring the fasting glucose level. Assays were carried out after 12 h of overnight fasting. The TT, mFG, HOMA-IR, and fasting insulin levels were higher in the PCOS group than that in the control group (Additional file 1: Table S1). However, BMI and age were comparable between the groups. The patient exclusion criteria for both groups were as follows: ovarian, adrenal, endometrial, cervical, and breast neoplasms, pelvic endometriosis, congenital adrenal hyperplasia, clinically and/or laboratory-confirmed endocrine disease (thyroid dysfunction, acromegaly, gigantism, or Cushing disease), diabetes type I or II, hyperprolactinemia, and unexplained vaginal bleeding. Ovarian cuneiform resection samples were collected during laparoscopic surgery, protected against RNA degradation by mixing with RNA later (Life Technologies), snap-frozen in liquid nitrogen, and stored at − 80 °C until analyzed.

### Isolation of human granulosa cells (GCs)

GCs were collected from 3 PCOS patients and 3 non-PCOS volunteers. Briefly, GCs were isolated from the preantral follicles of approximately 10–12 d postpartum ovaries via centrifugation at 1875 g (room temperature) for 10 min in tubes containing 80% Percoll; GCs formed a layer on the Percoll solution. GCs were cultured in DMEM/F12 (1:1, Gibco, Thermo Fisher Scientifc, Inc.) containing 10% fetal bovine serum (FBS, Sigma-Aldrich) for 3 days prior to the experiments. There was no significant difference in age between the patient and control groups. The present study was approved by the approval of the local research ethics committee of Qinghai Provincial People’s Hospital.

The article "MiR-140 targets RAP2A to enable the proliferation of insulin-treated ovarian granulosa cells" was retracted in 2023. Reasons: duplicated images; signs of a paper mill; unreliable results or conclusions.

### In vitro granulosa cell culture

All animal studies were approved by the Institutional Animal Care and Use Committee of the Qinghai Provincial People’s Hospital. The development of ovarian follicles was stimulated in 19-day-old female CFI mice by *i.p.* injection of equine chorionic gonadotropin (5 IU; eCG; FSH analog; Calbiochem, San Diego, CA). At 48 h post eCG injection, the mice were injected with hCG (5 IU; LH analog; Sigma, St. Louis, MO) to promote ovulation and luteinization. The ovaries were collected after 48 h post hCG injection. Through follicular puncture in PBS (containing 1 mM KH_2_PO_4_, 155 mM NaCl, 3 mM Na_2_HPO_4_, 10,010,049, Gibco™), we collected the granulosa cells from the ovarian tissues. The isolated granulosa cells were used for protein analysis, as well as for evaluating the gene expression and apoptosis (2.5 × 10^4^ cells/well in six-well fibronectin-coated tissue culture plates). Prior to cell culture, expression levels were determined in granulosa cells by RT-PCR. DMEM medium/F12 supplemented with gentamicin (1%) and fetal bovine serum (10%) was used for cell culture (5% CO_2_; 37 °C).

Cells were seeded in 6-well plates (ThermalFisher), and then treated with rh-insulin (Roche Diagnostics) at a concentration of 100 ng/ml for 24 h [8].

### miRNA array

The phenol-chloroform method (TRIzol; Invitrogen) was used to extract total RNA. Capillary electrophoresis was used to evaluate the RNA quality. The NEBNext Multiplex Small RNA Library Prep Set from Illumina (New England BioLabs, Inc., Ipswich, MA, USA) was used to prepare libraries for small RNA sequencing. The Agilent Bioanalyzer 2100 system was used for library quantification and the Fast QC quality control tool was used for quality control analysis of the raw sequence files. Adaptors were removed using Cutadapt (version 1.2.1). The data of poor quality were eliminated by trimming the sequences of lower quality. Based on clean reads, the miRNA was recognized at 21–22 nt (length) and Bowtie software (version 2; CGE Risk Management Solutions B.V., Leidschendam, The Netherlands) was used to identify the reference sequence. The analysis of novel miRNA functions was performed using the miRDeep2 software (version 2.0.0.8). The statistical significance in detected alterations was assessed by calculating the differential expression between the case and control specimen miRNAs.

The article "MiR-140 targets RAP2A to enable the proliferation of insulin-treated ovarian granulosa cells" was retracted in 2023. Reasons: duplicated images; signs of a paper mill; unreliable results or conclusions.

### Transfections

Cells were transfected with inhibitor of either miR-140 (5′-CAG UGG UUU UAC CCU AUG GUA G-3′), or NC inhibitor (5′-UCA CAA CCU CCU AGA AAG AGU AGA-3′), or miR-140 mimic (5′-CAG UGG UUU UAC CCU AUG GUA G-3′) or NC mimic (5′- UUG UAC UAC ACA AAA GUA CUG-3′) (RiboBio, Guangzhou, China) at 100 nM concentration using Lipofectamine 2000 reagent (Invitrogen) according to the manufacturer’s protocol.

### MTT assay

Cell viability was studied using MTT assay. Briefly, the collected cells were treated with 20 μL of MTT (0.5 mg/mL, m6494, Invitrogen™). The supernatant was discarded, and then 150 μL DMSO was added. Subswequently, absorbance was measured at 490 nm using an Infinite M200 microplate reader (provided by Tecan, Männedorf, Switzerland). Data from the MTT assays were analyzed by ANOVA analysis.

### EdU incorporation assay

Cell proliferation was studied using an EdU incorporation assay. Cells were seeded into 6-well plates. An EdU (A10044, Invitrogen™) stock solution in PBS (10 mg/mL) was diluted 1000× with the culture media 48 h post transfection. This was followed by a 60-min incubation with EdU. Next, the cells were fixed for 20 min using 4% paraformaldehyde, and permeabilized for 10 min with 0.3% Triton X-100. EdU incorporation was detected by Click-IT EdU Assay according to the manufacturer’s instructions (Invitrogen). The cells were examined under a fluorescence microscope (Olympus 600 auto-biochemical analyzer). Image analysis was performed using Image-Pro Plus software. Ten fields at 20 X magnification were obtained to evaluate the incorporation of EdU. DAPI positive cells were counted as total cells, while EdU stained cells was counted as EdU positive cells.

### Evaluation of cell apoptosis

Annexin V-FITC and PI apoptosis detection kit (V13242, Invitrogen™) were used to detect cell apoptosis. The collected cells were transfected, followed by resuspension in 20 μL of binding buffer and 20-min incubation using PI (5 μL) and annexin V-FITC (10 μL) in the dark. Cell death was estimated using flow cytometry (FC).

### Western blotting (WB)

Cells were lysed in RIPA buffer (150 mM NaCl, 50 mM Tris-HCl, 0.1% SDS, 1% NP-40, pH 7.2) having a mixture of protease inhibitor cocktail (Roche Applied Science). Protein quantification was done using a BCA Protein Quantitation Kit. After separation using SDS-PAGE (10%; Bio-Rad, CA, USA), the proteins were transferred to a PVDF membranes (provided by Millipore, MA, America; 0.45-μm). After 60-min blocking at 25 °C using 5% BSA, the membranes were incubated at 4 °C with the indicated primary antibody overnight. The primary antibody against: RAP2A (ab49685, Abcam, 1:1000), AKT (ab8805, Abcam, 1:1000) [45], phosphor AKT (ab38449, Abcam, 1:1000) [46], and GAPDH (ab8245, Abcam, 1:2500) were used. Subsequently, a 60 min of incubation of the membranes at 25 °C was done with the goat anti-rabbit/mouse IgG secondary antibodies, as appropriate. Immunoreactivity was measured using a Super Signal West Femto Maximum Sensitivity Substrate Kit (Thermo) on a C-DiGit Blot Scanner. The band density was analyzed and quantitated by Photoshop CS6 software.

The article "MiR-140 targets RAP2A to enable the proliferation of insulin-treated ovarian granulosa cells" was retracted in 2023. Reasons: duplicated images; signs of a paper mill; unreliable results or conclusions.

### RNA isolation and quantitative PCR (qPCR)

After sample preparation, Trizol reagent (Invitrogen, CA, USA) was used for the extraction of total RNA from cells. MiR-140 and RAP2A quantification was performed in a Roche Light-Cycler 480 Real-Time PCR system (Roche, Germany) using SYBR Green. GADPH was used as an internal reference. The SYBR Green PCR Master Mix was used to conduct qPCR on a Light Cycler 480 instrument, with the terminal volume adjusted at 20 μL, at the following PCR conditions- 95 °C for 10 min; followed with 40 cycles of the following: 95 °C for 15 s, 60 °C for 30 s, and 72 °C for 30 s. Target values were calculated based using the 2^-ΔΔCT^ method via normalization to the internal reference (GAPDH) relative to the calibrator (mean of the control samples). The specificity of qPCR amplification was verified by performing a melting curve analysis and agarose gel electrophoresis. Each sample in every group was measured in duplicate.

### Dual-luciferase reporter assay (DLRA)

DLRA was performed using RAP2A as the target. The entire RAP2A 3′-UTR region (5′-AGT GTC ACT TAA AGA ATC CAC-3′) was amplified and then inserted into PCGF1 plasmid. Site-directed mutagenesis was performed to eliminate the predicted miR-140 binding sites in the RAP2A gene. Cells expressing the mutant RAP2A 3′-UTR region (5′-GCT AGA CTT TAA AGA ATC CAC-3′) served as the control. The efficiency of transfection was monitored using a reporter control, i.e., the Renilla luciferase plasmid harboring the thymidine kinase promoter (pRL-TK vector, TaKaRa, Japan). HEK293T cells were co-transfected with miR-140 suppressor RAP2A-WT/MU or the miR-140/NC mimic via a luciferase reporter vector, after which DLRA was performed. HEK293T cells (commercially available from the Basic Research Institute of Peking Union Medical College Hospital) were cultivated in DMEM containing 10% FBS supplemented with mycillin. Cell incubation was conducted with 5% CO_2_ at 37 °C, and the culture media was replaced every other day. The cells were digested with tryptase (0.25%) between passages and were sub-cultured at 70 to 80% confluency.

The article "MiR-140 targets RAP2A to enable the proliferation of insulin-treated ovarian granulosa cells" was retracted in 2023. Reasons: duplicated images; signs of a paper mill; unreliable results or conclusions.

### RNA silencing

ShRNAs against RAP2A were used to reduce their expression. The shRNA targeting RAP2A (5′-AUA UCU ACA UGC ACU UCG GTT-3′) used in this study was designed and produced by Ruibiotech Co. (Beijing, China). 100 μM shRNA was added into 5 μL of RNase-free water. This was followed by the addition of transfection reagent (10 μL), and 15 min incubation at 25 °C. In this study, shRNA transfection of cells was conducted 24 h.

### Statistical analysis

Data are represented as mean ± SD. The differences between multiple groups or two groups were assessed using one-way ANOVA with Tukey post hoc test or a two-tailed Student’s *t*-test, respectively. *P* < 0.05 indicates statistical significance.

## Supplementary information

**Additional file 1: Table S1.** Anthropometric, metabolic and hormonal characteristics of the subjects.

## Data Availability

Not applicable.
